The article "Effect of Enhanced Recovery after Surgery with Integrated Traditional Chinese and Western Medicine on Postoperative Stress Response of Patients with Gastrointestinal Tumors" was published in 2022. Journal: Comput Math Methods Med.

# Effect of Enhanced Recovery after Surgery with Integrated Traditional Chinese and Western Medicine on Postoperative Stress Response of Patients with Gastrointestinal Tumors

**DOI:** 10.1155/2022/3663246

**Published:** 2022-07-08

**Authors:** Haiping Zhao, Wenhui Sun

**Affiliations:** Department of General Surgery, The First People's Hospital of Fuyang, Hangzhou, Zhejiang, China

## Abstract

**Objective:**

To investigate the effect of enhanced recovery after surgery (ERAS) with integrated traditional Chinese and Western medicine on postoperative stress response of patients suffering from gastrointestinal tumors.

**Methods:**

A total of 74 patients with gastrointestinal tumors who underwent surgical treatment in our hospital from April 2019 to March 2021 were recruited and randomized into the control group and the observation group (1 : 1). The control group received routine treatment and care, while the observation group received ERAS plus integrated traditional Chinese and Western medicine. Clinical observation was performed regarding changes in preoperative mood and postoperative pain level in each group. Changes in expression levels of plasma cortisol, C-reactive protein (CRP), interleukin-6 (IL-6), interleukin-8 (IL-8), and tumor necrosis factor-*β* (TNF-*β*) before and after surgery were detected in each group. Time of patients' first fart and defecation and complications after surgery in each group were recorded.

**Results:**

The visual analogue scale (VAS) of patients in the observation group after 12 and 24 h of surgery was significantly lower than that in the control group (12 h: observation group 2.0 (1.00, 3.00) vs. control group 4.00 (3.00, 5.00), *p* = 0.001; 24 h: observation group 2.00 (1.00, 3.00) vs. control group 3.00 (2.00, 5.00), *p* = 0.005). The preoperative anxiety degree of patients in the two groups was not statistically significant (*p* = 0.489). The plasma cortisol level of patients in the observation group after 24 and 48 h of surgery was significantly lower than that in the control group (24 h: observation group 426.54 ± 52.15 nmol/L vs. control group 508.32 ± 41.08 nmol/L, *p* = 0.001; 48 h: observation group 287.19 ± 44.24 nmol/L vs. control group 362.57 ± 43.46 nmol/L, *p* = 0.001). Patients' postoperative CRP, IL-6, IL-8, and TNF-*β* expression levels in the observation group were remarkably lower than those in the control group at all time points. The first postoperative defecation came earlier in the observation group than that in the control group (observation group 76.00 h (64.50, 87.50) vs. control group 89.00 h (73.50, 116.00), *p* = 0.007). There was 1 postoperative urinary tract infection in the observation group and 1 postoperative intestinal obstruction and 1 incisional wound infection in the control group.

The article "Effect of Enhanced Recovery after Surgery with Integrated Traditional Chinese and Western Medicine on Postoperative Stress Response of Patients with Gastrointestinal Tumors" was published in 2022. Journal: Comput Math Methods Med.

**Conclusion:**

ERAS with integrated traditional Chinese and Western medicine could effectively reduce the postoperative stress response and inflammatory reaction in patients with gastrointestinal tumors, contributing to the safe and quick recovery of gastrointestinal functions of patients.

## 1. Introduction

Gastrointestinal tumors are the most common type of malignant tumors in the stomach or intestines and include gastric cancer and colorectal cancer. Gastric cancer is the fifth most prevalent malignancy worldwide and can be divided into Epstein-Barr virus- (EBV-) positive subtype, Microsatellite Instability (MSI) subtype, Genomically Stable (GS) subtype, and Chromosomal Instability (CIN) subtype, according to the latest research of The Cancer Genome Atlas (TCGA) [1]. Chronic inflammation of the stomach is considered one of the risk factors for gastric cancer and may progress through steps encompassing atrophic gastritis, intestinal metaplasia, and dysplasia [2]. Colorectal cancer is the third major cancer in the digestive system and the fourth leading cause of cancer death in the world [3]. Its heritability is approximately 35% (95% confidence interval: 10%-48%) [4, 5]. Surgical resection is thought of as the only treatment regimen that can cure gastric cancer and colorectal cancer completely [6, 7]. Tumor resection and clearance of surrounding lymph nodes are the basis of surgical regimens for both gastric cancer and colorectal cancer [8]. Nevertheless, surgical injury triggers new problems like stress response.

Gastrointestinal tumor surgery features large surgical trauma, evident stress response, serious postoperative pain, and great risks for various postoperative complications [9]. All these postoperative traumas and stress responses prolong hospital days and increase treatment cost [9]. Systematic stress responses arising from surgical traumas mainly include neuroendocrine disorder and abnormal metabolisms. A relevant study elaborated that abdominal surgery will cause the abnormal activation of the Hypothalamic-Pituitary-Adrenal (HPA) axis and disrupt the normal circadian rhythm of cortisol secretion [10]. After a few hours of surgery, total plasma cortisol concentration had 4-fold elevation in relation to the normal level and reached peak [10]. Besides, high circulating levels of cortisol may directly result in organ damages [11]. In addition, a study illustrated that some serum cytokines such as interleukin-1 (IL-1), interleukin-6 (IL-6), and tumor necrosis factor-*β* (TNF-*β*) are related to abnormal secretion of plasma cortisol, and the expression level of these cytokines elevates after surgery [12]. Reducing stress response which is caused by surgical trauma and severity of neuroendocrine disorder or abnormal metabolisms can shorten patients' recovery after surgery, improve patients' life quality, and decrease the incidence of complications during the perioperative period.

The article "Effect of Enhanced Recovery after Surgery with Integrated Traditional Chinese and Western Medicine on Postoperative Stress Response of Patients with Gastrointestinal Tumors" was published in 2022. Journal: Comput Math Methods Med.

Enhanced recovery after surgery (ERAS) refers to a series of optimized perioperative measures based on evidence-based medicine taken by a team consisting of surgeons, anesthetists, and nurses [13, 14]. This measure is aimed at reducing physical and psychological traumatic stress of patients with surgery and help patients recover rapidly [13, 14]. ERAS can quicken postoperative recovery without increasing complication incidence [15]. A meta-analysis of gastric cancer showed that the C-reactive protein (CRP) level is significantly declined in patients applying ERAS after 3/4 and 7 days of surgery [16]. Furthermore, the IL-6 level is declined after 1 and 3/4 days of surgery, and the TNF-*α* level is also declined after 3/4 day of surgery [16]. Gustafsson et al. [17] researched 911 patients who received surgery for colon carcinoma. They discovered that risk of 5-year cancer-specific death of patients whose compliance to ERAS intervention ≥ 70% is decreased by 42% compared with other patients. In view of these findings, application of ERAS may help patients shorten the perioperative period and quickly recover.

Traditional Chinese Medicine (TCM) is a repository of experience in improving postoperative recovery effect. Auricular point sticking and TCM plaster are characteristic techniques of TCM and widely used in clinics for convenience and low cost. Owing to the connection of the pain center and auditory center in the cerebral cortex, the auditory center can be stimulated by auricular acupressure, then effectively inhibit the adjacent pain center to relieve pain [18]. Meanwhile, the mechanism regulates the excitement and inhibition of the cerebral cortex and autonomic nerve center under the cerebral cortex to diminish inflammation, relieve pain, and soothe nerves [19]. Auricular point sticking can improve postoperative gastrointestinal function recovery and is relevant to somatostatin downregulation and motilin elevation [20]. Despite the increasing number of relevant studies, little is reported about the effect of ERAS with integrated TCM and Western medicine on postoperative stress response of patients with gastrointestinal tumors.

This study is aimed at exploring the effect of routine care with ERAS plus integrated TCM and Western medicine on mood change, postoperative pain, gastrointestinal function recovery, and inflammatory reaction indicators of patients with gastrointestinal tumors.

The article "Effect of Enhanced Recovery after Surgery with Integrated Traditional Chinese and Western Medicine on Postoperative Stress Response of Patients with Gastrointestinal Tumors" was published in 2022. Journal: Comput Math Methods Med.

## 2. Materials and Methods

### 2.1. Data Sources and Patients' Inclusion Criteria

#### 2.1.1. Data Sources

Patients who underwent surgery for gastrointestinal tumors from April 2019 to March 2021 in First People's Hospital of Fuyang were selected as the study objects. All patients were diagnosed with gastrointestinal tumors by medical iconography and pathology. Patients who met the following criteria were excluded: (i) patients who had received chemotherapy or radiation before surgery; (ii) patients with cardiovascular, liver, kidney, brain, lung, or other serious diseases or patients with basic diseases like hypertension, diabetes, and mental illness; (iii) patients who had severe complications during the perioperative period and transferred to the intensive care unit; and (iv) patients during pregnancy or lactation. A total of 74 patients were finally included in this study and equally divided into the control group and observation group (37 patients for each group) according to different treatment and care regimens during the perioperative period. Patients' detailed baseline characteristics are shown in Table 1. Informed consent of patients was not included because it was a retrospective study. The presented study had been approved by the ethics committee of our hospital.

### 2.2. Research Methods

#### 2.2.1. Intervention

- *Basic treatment*. Patients in two groups both were given basic treatment. Patients' cardiomotility was monitored by electrocardiogram. Water and electrolyte were given to maintain acid-base balance. Intravenous nutrition was given during the period of fasting. Antibodies were also applied.
- *Treatment or Care Plan for the Control Group*. Treatment or care plan for the control group includes routine treatment or care only.

*Western medicine intervention*: (a) surgical plan and risk were explained to patients before surgery. The fasting started 10 h before surgery. Water deprivation began 6 h before surgery. Routine bowel preparation was performed. (b) Two drainage tubes were placed during surgery and were removed after 7-9 d of surgery. Intraoperative thermal insulation was not emphasized. (c) Patient-Controlled Intravenous Analgesia (PCIA) and opioid drugs were used after surgery to relieve pain. Patients were allowed to drink water and eat after intestinal ventilation. (d) The catheter was removed after 2 d of surgery. (e) Patients were not guided to get early ambulation.

(iii) *Treatment or Care Plan in the Observation Group*. The treatment plan in the observation group contained Western medicine intervention and TCM medicine intervention.

The article "Effect of Enhanced Recovery after Surgery with Integrated Traditional Chinese and Western Medicine on Postoperative Stress Response of Patients with Gastrointestinal Tumors" was published in 2022. Journal: Comput Math Methods Med.

*Western medicine intervention*: (a) ERAS-related concepts, measures, surgical plan, and risk were explained to patients before surgery. (b) 1000 mL 10% glucose solution was given to patients 10 h before surgery. 500 mL 10% glucose solution was given to patients 2 h before surgery. Routine bowel preparation was not performed. (c) A drainage tube was placed during surgery and removed after 3-5 d of surgery. Gastric tubes were not routinely placed in principle (or removed after 24 h of surgery if placed). Thermal insulation was emphasized during surgery. (d) PCIA and nonsteroidal anti-inflammatory drugs (by oral) were used to relieve pain. Opioid drug use was reduced. (e) Water drinking and liquid diet were allowed on the day of surgery. (f) The catheter was removed after 24 h of surgery. (vii) Early ambulation was guided, including performing a semireclining position and turn-over after postoperative awakening from anesthesia, standing near the bed or walking under assistance after 18-24 h of surgery, indoor activities under assistance after 24-36 h of surgery, and walking in the corridor out of the ward and washing by themselves under assistance after 48 h of surgery. Activity amount and time increased gradually without making patients feel tired.

*TCM intervention*: (a) TCM plaster was given to patients: 300 g Sargentodoxa, 300 g rheum, 300 g salvia, 200 g fructus, 150 g officinal magnolia bark, and 75 g fructus Evodiae were quickly washed and dried in a drying oven at 50°C low temperature. After mixing, medicines were ground to superfine powder in 100,000 mesh size for 1 h. Then, the medicines were packed as powder bags (8.0 g/bag) by using a powder packing machine in the clean zone. Next, the powder was placed into plasters, fixed, and sealed to make TCM plasters. The TCM plaster was used immediately after surgery by sticking on the center of the abdomen taken navel (Shenque acupoint). The plaster was changed at 4:00 pm every day from the first day after surgery, and this procedure was repeated for 7 d. (b) Auricular acupoint sticking: this was conducted within 0.5 h after patients returned to the ward. That was to say, after being routinely disinfected with 75% alcohol wipes, patients' auricular acupoints (Shenmen, subcortical auricular point, endocrine auricular point) were accurately fixed with wangbuliuxing seed auricular acupoint sticking. The sticking was pressed with the index finger and thumb. Each acupoint was pressed for 1 min a time and repeated every 15 min. The pressing was undertaken on two ears in the meanwhile from gentle to heavy until the patient felt distension, acid, and radiation. This process was performed three times a day for 2 successive days.

The article "Effect of Enhanced Recovery after Surgery with Integrated Traditional Chinese and Western Medicine on Postoperative Stress Response of Patients with Gastrointestinal Tumors" was published in 2022. Journal: Comput Math Methods Med.

#### 2.2.2. Observation Indexes, Time, and Methods

*(1) Main Outcome Indexes*.

- The visual analogue scale (VAS) is a validated subjective measure of acute and chronic pain to document patients' pain progression or to compare pain severity in patients with similar conditions [21]. Basically, it uses a vernier scale about 10 cm in length. On the one side, there are “0” and “10” at both ends and 10 marks in between. 0 score indicates no pain, and 10 scores represent unbearable severe pain.

VAS was conducted on patients after 3, 6, 12, 24, and 48 h of surgery to evaluate the pain when patients rested and positively coughed.

(b) Stress response index: plasma cortisol changes were measured before surgery and after 3, 24, and 48 h of surgery. At each time point, venous blood was collected from the antecubital vein to the heparin anticoagulant tube, centrifuged at 3,000 rpm for 5 min, and then preserved at 4°C until use
(c) Inflammatory factor index: changes in CRP, IL-6, IL-8, and TNF-*β* levels were measured before surgery and after 3, 24, and 48 h of surgery. At each time, venous blood was collected from the antecubital vein to the heparin anticoagulant tube, centrifuged at 3,000 rpm for 5 min, and then preserved at 4°C until use

*(2) Secondary Outcome Indexes*.

- Self-rating anxiety scale (SAS): patients' anxiety was determined by SAS designed by Zung [22] at enrollment and when entering the operating room. There were 20 items in SAS (including 5 reverse coded items) with each item having 4 choices scoring from 1 to 4. Scores of the 20 items were added and then multiplied by 1.25 to select the integer part as the standard scores. According to results of the Chinese national norm, a standard score < 50 refers to no anxiety, 50 ≤ standard score < 60 refers to mild anxiety, 60 ≤ standard score < 70 refers to moderate anxiety, and standard score ≥ 70 refers to severe anxiety [23]
- Gastrointestinal function recovery: first time to fart and defecate after surgery
- Postoperative complication incidence rate and hospitalization expense

#### 2.2.3. Discharge Criteria and Follow-Up Visit

- Discharge criteria: unified discharge criteria were applied to two groups. Details were shown as follows: (a) complete recovery of oral feeding and no need for intravenous infusion, (b) no drainage or decompression tubes required, (c) simple off-bed activities were available, and (d) patients who were evaluated to be able to be discharged to leave the hospital according to their willingness
- Follow-up: all patients were followed up for 6 m by outpatient follow-up and telephone follow-up. Complications were recorded

### 2.3. Statistical Analysis

SPSS 23.0 and Prism 8.0 were applied for statistical analysis. Measurement data were shown as the mean ± standard deviation (SD) or *M* (P25, P75). Enumeration data were shown as the percentage (%). *T* test or *U* test was applied for comparison of measurement data between groups. The Chi-squared test or Fisher's exact test was applied for comparison of enumeration data between groups. *p* < 0.05 indicated that the difference between groups was statistically significant.

The article "Effect of Enhanced Recovery after Surgery with Integrated Traditional Chinese and Western Medicine on Postoperative Stress Response of Patients with Gastrointestinal Tumors" was published in 2022. Journal: Comput Math Methods Med.

## 3. Results

### 3.1. Patients' Clinical Baseline Level

For the control group, average age was 46.49 ± 9.57, there were 16 men and 21 women, the weight index was 21.74 ± 1.66, 10 patients had a smoking history, 22 patients were diagnosed with gastric cancer, 15 patients were diagnosed with colorectal cancer, 18 patients were in I stage, and 19 patients were in II stage.

For the observation group, average age was 47.65 ± 10.04, there were 21 men and 16 women, the weight index was 22.08 ± 1.51, 10 patients had a smoking history, 16 patients were diagnosed with gastric cancer, 21 patients were diagnosed with colorectal cancer, 23 patients were in I stage, and 14 patients were in II stage.

Differences in each baseline characteristic (Table 1) between groups had no statistical significance (*p* > 0.05), and the factors were comparable.

### 3.2. Main Outcome Indexes

Patients' postoperative pain degree in two groups was assessed by VAS. The pain degree in the two groups both elevated first and then declined. The pain degree of patients in the observation group was lower than that of the control group after 12 h (2.00 (1.00, 3.00) vs. 4.00 (3.00, 5.00), *p* = 0.001) and 24 h (2.00 (1.00, 3.00) vs. 3.00 (2.00, 5.00), *p* = 0.005) of surgery (Figure 1(a)).

Changes in patients' stress response in two groups were evaluated by plasma cortisol concentration. The plasma cortisol concentration of patients in the two groups both reached the peak after 24 h of surgery (control group: 508.32 ± 41.08 nmol/L vs. observation group: 426.54 ± 52.15 nmol/L, *p* = 0.001) and then declined after 24-48 h of surgery (control group: 362.57 ± 43.46 nmol/L vs. observation group: 287.19 ± 44.24 nmol/L, *p* = 0.001) (Figure 1(b)).

These results suggested that the treatment and care of integrating traditional Chinese and Western medicine with ERAS reduced patients' pain levels and plasma cortisol levels in comparison with conventional treatment and care.

Afterwards, the expression level of CRP, IL-6, IL-8, and TNF-*β* of patients in each group before and after surgery was detected. CRP of patients in two groups continuously elevated after surgery (Figure 2(a)), while the elevation trend in the observation group weakened after 48 h of surgery (control group: 187.35 ± 15.97 mg/L vs. observation group: 171.65 ± 19.67 mg/L, *p* = 0.001). The IL-6 expression level of patients in two groups presented a statistically significant difference after 3 h (control group: 95.16 ± 23.63 pg/L vs. observation group: 78.57 ± 20.97 pg/L, *p* = 0.005), 24 h (control group: 112.03 ± 24.66 pg/L vs. observation group: 94.19 ± 32.57 pg/L, *p* = 0.018), and 48 h (control group: 123.03 ± 28.59 pg/L vs. observation group: 105.78 ± 33.42 pg/L, *p* = 0.038) of surgery (Figure 2(b)). The IL-8 expression level of patients in two groups continuously elevated within 24 h after surgery while declined during 24-48 h after surgery and showed a statistically significant difference after 48 h (control group: 48.76 ± 3.63 pg/L vs. observation group: 41.92 ± 5.83 pg/L, *p* = 0.001) (Figure 2(c)). The TNF-*β* expression level of patients in two groups started to decline after 3 h of surgery (Figure 2(d)). The declined trend of TNF-*β* expression level after 24 h (control group: 1994.38 ± 220.75 pg/L vs. observation group: 1634.38 ± 185.40 pg/L, *p* = 0.001) and 48 h (control group: 1452.22 ± 200.29 pg/L vs. observation group 1230.54 ± 100.13 pg/L, *p* = 0.001) of surgery was more significant in the observation group than the control group. In conclusion, the postoperative CRP, IL-6, IL-8, and TNF-*β* levels of patients in the observation group were remarkably lower than those in the control group at different time points.

The article "Effect of Enhanced Recovery after Surgery with Integrated Traditional Chinese and Western Medicine on Postoperative Stress Response of Patients with Gastrointestinal Tumors" was published in 2022. Journal: Comput Math Methods Med.

### 3.3. Secondary Outcome Indexes

The patients' psychological anxiety degree at enrollment and when entering the operating room in each group was evaluated by Zung's SAS. Interestingly, it disclosed that patients in the observation group had more significantly severe anxiety at enrollment (control group: 32.00 (25.00, 44.00) vs. observation group: 39.00 (30.00, 48.50), *p* = 0.015). Patients' first postoperative defecation time in the observation group was earlier than that in the control group (control group: 89.00 h (73.50, 116.00) vs. observation group: 76.00 h (64.50, 87.50), *p* = 0.007). Patients' hospitalization expense in the observation group was significantly lower than that in the control group (control group: 61365 ± 5840 RMB vs. observation group: 57607 ± 6801 RMB, *p* = 0.013). In conclusion, the observation of postoperative defecation time and hospitalization costs was superior to the control group. A specific comparison of secondary outcome indexes is shown in Table 2.

### 3.4. Postoperative Complications

We performed a 6-month follow-up visit on patients in each group and recorded their complications during the period, as shown in Table 3. There was 1 case of postoperative intestinal obstruction and 1 case of postoperative incision infection in the control group. In the observation group, there was 1 case of postoperative urinary tract infection. Postoperative complications were less developed in both groups.

The article "Effect of Enhanced Recovery after Surgery with Integrated Traditional Chinese and Western Medicine on Postoperative Stress Response of Patients with Gastrointestinal Tumors" was published in 2022. Journal: Comput Math Methods Med.

## 4. Discussion

ERAS has been widely applied in the postoperative recovery of tumor surgery, such as liver resection for hepatocellular carcinoma [24], esophagectomy [25], pulmonary lobectomy for lung cancer [26], gastrectomy for gastric cancer [27], and colorectal cancer surgery [28]. Besides, a study on Japanese patients indicated that ERAS can help colorectal cancer patients rapidly recover, and the postoperative hospitalization time of patients who applied ERAS was evidently shorter than that of patients in the control group [29]. However, the study did not compare the indexes including patients' postoperative stress response and inflammatory factors in two groups; therefore, the results were relatively simple [29]. Another study about the recovery of patients who received gastrectomy and applied ERAS found that patients in the ERAS group recovered normal diet more quickly than patients in the control group [30]. This study combined TCM methods on the basis of ERAS and explored the effect of ERAS with integrated TCM and Western medicine on postoperative stress response of patients with gastrointestinal tumors.

This study assessed patients' postoperative pain degree in two groups through VAS. The pain degree within 6 h after surgery both elevated. As time passed, the pain degree of patients in the observation group was significantly weaker than that in the control group. Moreover, the effect of ERAS plus integrated TCM and Western medicine on postoperative stress response was evaluated by the plasma cortisol level of patients in each group. A relevant study revealed that following colorectal carcinoma resection, the patients' plasma cortisol level elevates on d 1 and 5 after surgery, while the level of patients who applied ERAS only elevates on day 5 after surgery, suggesting that ERAS can help patients reduce stress response [31]. Our study demonstrated that the postoperative plasma cortisol level of patients in the observation group who received ERAS with integrated TCM and Western medicine recovered to the normal level more quickly than that in the control group. The inflammatory index of patients in each group was also compared in this study. A relevant study illustrated that ERAS could make inflammatory-related factors recover to a normal level more quickly, and the CRP level was lower than that in the control group [32]. Our study manifested that CRP of patients in two groups within 48 h after surgery continuously elevated, and the elevation slowed then in the observation group. After 48 h of surgery, the CRP level of patients in the observation group was significantly lower than that in the control group, and the difference exhibited a statistical significance. A study detected the IL-6 level of patients in the ERAS group and the control group after colorectal cancer surgery, and it was disclosed that the IL-6 level in the ERAS group after 1, 3, and 5 d of surgery was lower than that in the control group [33]. Similarly, it was discovered here that the postoperative IL-6 level of patients in the observation group and control group continuously elevated, and overall, the IL-6 expression level of patients in the observation group was lower than that in the control group. Besides, the expression level of IL-8 and TNF-*β* was also detected. It was indicated that ERAS with integrated TCM and Western medicine could effectively reduce patients' postoperative inflammatory response.

The article "Effect of Enhanced Recovery after Surgery with Integrated Traditional Chinese and Western Medicine on Postoperative Stress Response of Patients with Gastrointestinal Tumors" was published in 2022. Journal: Comput Math Methods Med.

A study elaborated that the first defecation time of patients who underwent duodenectomy and received ERAS was 3 ± 2 days and was shorter than 4 ± 2 days of patients in the control group, exhibiting a statistically significant difference [34]. According to our study, it was discovered that ERAS with integrated TCM and Western medicine could effectively shorten postoperative first defecation time of gastrointestinal cancer patients. The time of patients in the observation group was significantly shorter than the time in the control group. In terms of safety, a relevant study showed that colorectal cancer patients in the control group and the ERAS group were both more likely to have intestinal obstruction [35]. We tracked postoperative complications of patients in each group and found that there was 1 postoperative intestinal obstruction and 1 postoperative incision infection in the control group and 1 postoperative urinary tract infection in the observation group. The overall postoperative complication incidence of patients in the two groups was relatively low, suggesting that ERAS with integrated TCM and Western medicine was safe to improve patients' postoperative recovery.

Taken together, this study investigated the effect of ERAS with integrated TCM and Western medicine on the stress response of patients with gastrointestinal tumors. According to the results of this study, it was believed that ERAS with integrated TCM and Western medicine could effectively and safely decline the postoperative stress response and inflammatory reaction of gastrointestinal tumor patients. Furthermore, patients' gastrointestinal functions could quickly recover.

## Figures and Tables

**Figure 1:** Changes in patients' preoperative and postoperative painful degree and plasma cortisol level in each group: (a) VAS scores compared changes in patients' postoperative pain degree in each group; (b) changes in patients' postoperative plasma cortisol level in each group. VAS: visual analogue scale; ^∗∗^*p* < 0.01, ^∗∗∗^*p* < 0.001.

The article "Effect of Enhanced Recovery after Surgery with Integrated Traditional Chinese and Western Medicine on Postoperative Stress Response of Patients with Gastrointestinal Tumors" was published in 2022. Journal: Comput Math Methods Med.

**Figure 2:** Patients' preoperative and postoperative inflammatory reaction-related indexes in each group: (a) patients' preoperative and postoperative CRP expression level in each group; (b) patients' preoperative and postoperative IL-6 expression level in each group; (c) patients' preoperative and postoperative IL-8 expression level in each group; (d) patients' preoperative and postoperative TNF-*β* expression level in each group. Abbreviations: CRP: C-reactive protein; IL-6: interleukin-6; IL-8: interleukin-8; TNF-*β*: tumor necrosis factor-*β*. ^∗^*p* < 0.05, ^∗∗^*p* < 0.01, and ^∗∗∗^*p* < 0.001.

**Table 1:** Patients' clinical baseline characteristics in each group.

Baseline characteristics	Group		*p* value
	Control group (37)	Observation group (37)	
Age (years)	46.49 ± 9.57	47.65 ± 10.04	0.612
*Gender*			0.353
Men (%)	16 (43)	21 (57)	
Women (%)	21 (57)	16 (43)	
Weight index	21.74 ± 1.66	22.08 ± 1.51	0.355
*Smoking history*			1.000
No (%)	27 (73)	27 (73)	
Yes (%)	10 (27)	10 (27)	
*Tumor type*			0.245
Gastric cancer (%)	22 (59)	16 (43)	
Colorectal cancer (%)	15 (41)	21 (57)	
*Tumor stage*			0.350
Stage I (%)	18 (49)	23 (62)	
Stage II (%)	19 (51)	14 (38)	

**Table 2:** Secondary outcome indexes.

Secondary indexes	Control group (*N* = 37)	Observation group (*N* = 37)	*p* value
*SAS score*			
Enrollment	32.00 (25.00, 44.00)	39.00 (30.00, 48.50)	0.015
Before operation	49.00 (39.50, 53.50)	48.00 (42.00, 55.00)	0.489
Postoperative first fart time (day)	39.00 (28.50, 46.50)	34.00 (30.50, 42.50)	0.372
Postoperative first defecation time (day)	89.00 (73.50, 116.00)	76.00 (64.50, 87.50)	0.007
Hospitalization expense (RMB)	61365 ± 5840	57607 ± 6801	0.013

Abbreviation: SAS: self-rating anxiety scale.

**Table 3:** Patients' postoperative complications in each group.

Postoperative complications	Control group (*N* = 37)	Observation group (*N* = 37)
Intestinal obstruction	1	0
Abdominal infection	0	0
Incision infection	1	0
Postoperative urinary tract infection	0	1
Total	2	1

## Data Availability

The data and materials in the current study are available from the corresponding author on reasonable request.

## References

[1] Seidlitz T., Chen Y. T., Uhlemann H. (2019). Mouse models of human gastric cancer subtypes with stomach-specific CreERT2-mediated pathway alterations. *Gastroenterology*.

[2] Yu G., Torres J., Hu N. (2017). Molecular characterization of the human stomach microbiota in gastric cancer patients. *Frontiers in Cellular and Infection Microbiology*.

The article "Effect of Enhanced Recovery after Surgery with Integrated Traditional Chinese and Western Medicine on Postoperative Stress Response of Patients with Gastrointestinal Tumors" was published in 2022. Journal: Comput Math Methods Med.

[3] Zhu L., Tong Y. X., Xu X. S., Xiao A. T., Zhang Y. J., Zhang S. (2020). High level of unmet needs and anxiety are associated with delayed initiation of adjuvant chemotherapy for colorectal cancer patients. *Support Care Cancer*.

[4] Song N., Lee J., Cho S., Kim J., Oh J. H., Shin A. (2019). Evaluation of gene-environment interactions for colorectal cancer susceptibility loci using case-only and case-control designs. *BMC Cancer*.

[5] Monahan K. J., Bradshaw N., Dolwani S. (2020). Guidelines for the management of hereditary colorectal cancer from the British Society of Gastroenterology (BSG)/Association of Coloproctology of Great Britain and Ireland (ACPGBI)/United Kingdom Cancer Genetics Group (UKCGG). *Gut*.

[6] Liu C. A., Huang K. H., Chen M. H. (2017). Comparison of the surgical outcomes of minimally invasive and open surgery for octogenarian and older compared to younger gastric cancer patients: a retrospective cohort study. *BMC Surgery*.

[7] Yang Z. F., Wu D. Q., Wang J. J., Lv Z. J., Li Y. (2018). Short- and long-term outcomes following laparoscopicvsopen surgery for pathological T4 colorectal cancer: 10 years of experience in a single center. *World Journal of Gastroenterology*.

[8] Salibasic M., Pusina S., Bicakcic E. (2019). Colorectal cancer surgical treatment, our experience. *Medical Archives*.

[9] Manou-Stathopoulou V., Korbonits M., Ackland G. L. (2019). Redefining the perioperative stress response: a narrative review. *British Journal of Anaesthesia*.

[10] Cerejeira J., Batista P., Nogueira V., Vaz-Serra A., Mukaetova-Ladinska E. B. (2013). The stress response to surgery and postoperative delirium. *Journal of Geriatric Psychiatry and Neurology*.

[11] Skovira E. J., Behrend E. N., Martin L. G., Palmer L. E., Kemppainen R. J., Lee H. P. (2017). Effect of laparotomy on the pituitary-adrenal axis in dogs. *American Journal of Veterinary Research*.

[12] Siekmann W., Eintrei C., Magnuson A. (2017). Surgical and not analgesic technique affects postoperative inflammation following colorectal cancer surgery: a prospective, randomized study. *Colorectal Disease*.

[13] Ljungqvist O., Scott M., Fearon K. C. (2017). Enhanced recovery after surgery. *JAMA Surgery*.

[14] Bardram L., Funch-Jensen P., Jensen P., Crawford M. E., Kehlet H. (1995). Recovery after laparoscopic colonic surgery with epidural analgesia, and early oral nutrition and mobilisation. *Lancet (London, England)*.

[15] Senturk J. C., Kristo G., Gold J., Bleday R., Whang E. (2017). The development of enhanced recovery after surgery across surgical specialties. *Journal of Laparoendoscopic & Advanced Surgical Techniques. Part A*.

The article "Effect of Enhanced Recovery after Surgery with Integrated Traditional Chinese and Western Medicine on Postoperative Stress Response of Patients with Gastrointestinal Tumors" was published in 2022. Journal: Comput Math Methods Med.

[16] Wee I. J. Y., Syn N. L., Shabbir A., Kim G., So J. B. Y. (2019). Enhanced recovery versus conventional care in gastric cancer surgery: a meta-analysis of randomized and non-randomized controlled trials. *Gastric Cancer*.

[17] Gustafsson U. O., Oppelstrup H., Thorell A., Nygren J., Ljungqvist O. (2016). Adherence to the ERAS protocol is associated with 5-year survival after colorectal cancer surgery: a retrospective cohort study. *World Journal of Surgery*.

[18] Gao S., Zhu Z., Han S. (2010). Effect of auricular plaster therapy combined with soothing touch on perioperative stress response of patients undergoing abdominal surgery. *Journal of emergency in traditional chinese medicine*.

[19] He Z., Liu G., Li X., Yao J. (2017). Clinical observation on the postoperative pain after cesarean section with the intervention of auricular point pressing combined with perioperative psychological nursing. *Shanxi Journal of Traditional Chinese Medicine*.

[20] Wei X., Qiu H., Zhang Q. (2014). Shenhuang powder paste for 110 patients with gastrointestinal dysfunction after abdominal surgery: a prospective multi-center randomized controlled clinical study. *Journal of Traditional Chinese Medicine*.

[21] Delgado D. A., Lambert B. S., Boutris N. (2018). Validation of digital visual analog scale pain scoring with a traditional paper-based visual analog scale in adults. *Journal of the American Academy of Orthopaedic Surgeons. Global research & reviews*.

[22] Dunstan D. A., Scott N. (2020). Norms for Zung's self-rating anxiety scale. *BMC Psychiatry*.

[23] Du Y., Cui Y., Cai X., Li Y., Yang D. (2020). Analysis of influencing factors of preoperative anxiety or depression in patients with lung cancer surgery. *Zhongguo Fei Ai Za Zhi*.

[24] Ren Q. P., Luo Y. L., Xiao F. M. (2020). Effect of enhanced recovery after surgery program on patient-reported outcomes and function recovery in patients undergoing liver resection for hepatocellular carcinoma. *Medicine (Baltimore)*.

[25] Kano K., Aoyama T., Maezawa Y. (2019). Postoperative level of C-reactive protein is a prognosticator after esophageal cancer surgery with perioperative steroid therapy and enhanced recovery after surgery care. *In Vivo*.

[26] Chen F., Wang G. (2020). Enhanced recovery after surgery for lung cancer patients. *Open Med (Wars)*.

[27] Cao S., Zheng T., Wang H. (2021). Enhanced recovery after surgery in elderly gastric cancer patients undergoing laparoscopic total gastrectomy. *The Journal of Surgical Research*.

[28] Gustafsson U. O., Hausel J., Thorell A. (2011). Adherence to the enhanced recovery after surgery protocol and outcomes after colorectal cancer surgery. *Archives of Surgery*.

The article "Effect of Enhanced Recovery after Surgery with Integrated Traditional Chinese and Western Medicine on Postoperative Stress Response of Patients with Gastrointestinal Tumors" was published in 2022. Journal: Comput Math Methods Med.

[29] Shida D., Tagawa K., Inada K. (2015). Enhanced recovery after surgery (ERAS) protocols for colorectal cancer in Japan. *BMC Surgery*.

[30] Desiderio J., Stewart C. L., Sun V. (2018). Enhanced recovery after surgery for gastric cancer patients improves clinical outcomes at a US cancer center. *Journal of gastric cancer*.

[31] Ren L., Zhu D., Wei Y. (2012). Enhanced Recovery After Surgery (ERAS) program attenuates stress and accelerates recovery in patients after radical resection for colorectal cancer: a prospective randomized controlled trial. *World Journal of Surgery*.

[32] Jaloun H. E., Lee I. K., Kim M. K. (2020). Influence of the enhanced recovery after surgery protocol on postoperative inflammation and short-term postoperative surgical outcomes after colorectal cancer surgery. *Annals of coloproctology*.

[33] Mari G., Crippa J., Costanzi A., Mazzola M., Rossi M., Maggioni D. (2016). ERAS protocol reduces IL-6 secretion in colorectal laparoscopic surgery: results from a randomized clinical trial. *Surgical Laparoscopy, Endoscopy & Percutaneous Techniques*.

[34] Deng X., Cheng X., Huo Z. (2017). Modified protocol for enhanced recovery after surgery is beneficial for Chinese cancer patients undergoing pancreaticoduodenectomy. *Oncotarget*.

[35] Shida D., Tagawa K., Inada K. (2017). Modified enhanced recovery after surgery (ERAS) protocols for patients with obstructive colorectal cancer. *BMC Surgery*.

